The article "Detection Rate and Prognosis of Lymph Nodes in Gastric Cancer Using Nano Carbon Combined with In Vitro Anatomical Sorting" was retracted in 2023. Reasons: suspected computer-generated content; unreliable results or conclusions; concerns about the data; concerns about the results or conclusions.

# Detection Rate and Prognosis of Lymph Nodes in Gastric Cancer Using Nano Carbon Combined with *In Vitro* Anatomical Sorting

**DOI:** 10.1155/2022/4540176

**Published:** 2022-08-23

**Authors:** Jun Ma, Chongren Ren, Gang Du, Jinxi Wang, Zhenguo Han, Huhu Li, Huiyu Li, Liang Xue

**Affiliations:** ^1^General Surgery Department, Shanxi Bethune Hospital, Shanxi Academy of Medical Sciences, Tongji Shanxi Hospital, Third Hospital of Shanxi Medical University, Taiyuan 030032, China; ^2^Tongji Hospital, Tongji Medical College, Huazhong University of Science and Technology, Wuhan 430030, China; ^3^Third Hospital of Shanxi Medical University, Shanxi Bethune Hospital, Shanxi Academy of Medical Sciences, Tongji Shanxi Hospital, Taiyuan 030032, China

## Abstract

In this study, we are going to investigate the effect of nano carbon combined with *ex vitro* anatomical sorting on the detection rate of lymph nodes (LNs) in gastric cancer (GC) along with the analysis of the correlation between LNs detection rate and patients' prognosis. The clinical data of patients undergoing radical gastrectomy in Shanxi Bethune Hospital, Shanxi Academy of Medical Sciences, Tongji Shanxi Hospital, Third Hospital of Shanxi Medical University from January 2018 to January 2019 were examined retrospectively. According to whether they adopt nano carbon tracing and specimen sorting method, patients were divided into nano carbon and control groups. The respective rate of detection and correlation of total and positive LNs, respectively, clinical treatment, tumor marker level, and long-term prognosis were matched between these groups. At the same time, the effects of the nano carbon tracer on the detection of total and positive LNs were evaluated. In nano carbon group, more LN specimens could be detected, and the number of positive LNs increased significantly. In addition, in patients with different infiltration stages and LN substations, more LNs could be detected in the nano carbon group for examination, and the detection rate of LNs with diameter less than 5 mm was also more. Furthermore, LNs (preferably positive in number) were correlated positively with the attained LNs number. Otherwise, the use of nano carbon suspension could better label LNs in each substation, especially N1 station, and improve micro-LN detection rate. At the same time, the positive metastasis rate in black-stained LNs was higher (31.67% vs. 13.51%). In relation to the clinical prognosis, CEA's level, i.e., CA199 and CA125, in the nano carbon group is controlled more effectively. Their condition was not easy to progress and relapse, and their mortality was further reduced. As a result, nano carbon, coupled with *ex vitro* anatomical sorting, may considerably enhance the detection rate of total and positive LNs, thereby improving the accuracy of clinical staging in GC patients, which has a good influence on their long-term prognosis.

## 1. Introduction

Gastric cancer (GC), specifically with the 5-year survival rate of only about 25% [1], is a common digestive tract's malignant tumor in China, and in approximately all tumors, the expected rate of its occurrence is ranked third. Currently, the incidence of GC has increased year by year because of poor living and eating habits, and tends to be younger, which will bring great challenges to China's healthcare system [2]. At present, among the various treatment methods of GC, surgical resection is still the main treatment method [3]. As lymph node (LN) metastasis often has occurred when patients visit, in addition to accurately completing the complete tumor resection, a thorough LN dissection is also the key point during the operation [4, 5]. LN detection rate is one of the effective indicators to evaluate surgery quality. It is also helpful to make accurate staging of patients' condition during clinical diagnosis and treatment [6]. Based on the effective statistics, it is stated that approximately every 10^th^ of the additional LNs has the capacity to effectively improve the rate of detection of metastatic LNs [7], which is of great significance to optimize the postoperative treatment plan and improve patients' prognosis. In addition, the increased number of negative LNs is also one of the factors affecting the prognosis of patients [8, 9]. Therefore, effectively improving the detection rate of LNs during the GC surgery has an important impact on accurate clinical staging, guiding clinical treatment, and prognosis judgment.

In the process of LN dissection, the LN metastasis pathway of GC is complex and multidirectional, and the blood vessels around the stomach are rich, which increase the risk and difficulty of complete LN dissection. Therefore, relying solely on experience and naked eye for LN dissection is easy to lead to the omission of smaller LNs, thus reducing LN detection rate. In this study, to enhance the display of precancerous associated LNs, we selected nano carbon as a tracer. After treatment with nanotechnology, nano carbon has a high tendency of lymphatic system [10]. The main reason is that the size of nano carbon particles can be adjusted to about 150 nm, which cannot effectively pass through the 30–50 nm gap of capillary endothelium, however, it can quickly pass through the 120–500 nm gaps of the lymphatic endothelial cells [11, 12]. As a result, nano carbon can effectively aggregate in lymphatic vessels, and the draining lymph nodes around the tumor can be effectively stained black. It has a significant tracing effect on SLN and regional LNs to effectively guide the scope of LN dissection and improve the LN detection rate [13].

On the premise of standardized D2 LN dissection, improving *ex vitro* LN sorting technology and optimizing the LN sorting method are the main factors affecting the detective number of LNs. In the sorting of isolated LN specimens, launching a special LN's sorting team and giving them theoretical learning and practical practice can be used as a supplement to surgical sorting for the improvement of the rate of the detection of LNs, more specifically, micro-LNs. Previous studies have shown that approximately 40 percent of metastatic LNs have a diameter less than 5 mm [14, 15], and these LNs are difficult to distinguish from the surrounding adipose tissue because of their small volume. Improving micro-LN detection rates is critical for accurately forecasting patient state and clinical staging.

Therefore, to address this issue, we have integrated nano carbon with the anatomical sorting of *ex vitro* in the LN dissection of GC patients and thoroughly examined its effect on LN's rate of detection and prognosis of patients. For this, we have divided these patients into two different groups as described above and examined them.

The remaining sections and its contribution are given below.

In the subsequent section, materials and methods, i.e., why the proposed problem is assumed and how it is resolved with the proposed approach, are described in detail. In section 3, the results and discussion on those results are presented, whereas the finalized remarks are presented in section 4, i.e., conclusion.

## 2. Materials and Methods

### 2.1. Research Object Selection

From Jan-2018 to Jan-2019, the clinical data of GC patients treated at Shanxi Bethune Hospital, Shanxi Academy of Medical Sciences, Tongji Shanxi Hospital, and Shanxi Medical University's Third Hospital were retrospectively evaluated. Criteria for entry: (1) stomach cancer was identified using the criteria outlined in “gastric cancer: ESMO clinical practice guidelines for diagnosis, therapy, and follow-up” [16]. (2) Age range: 18 to 60 years old, (3) having gastric cancer radical surgery, (4) no distant metastases were seen on preoperative CT and ultrasonic gastroscopy, (5) no radiation or immunotherapy was given before to the procedure, and (6) complete clinical data. Criteria for exclusion: (1) recurrent GC, (2) previous abdominal surgery, (3) combined with malignant tumors in other regions, (4) allergic to the medications used in this study, and (5) combined with severe cardiovascular and cerebrovascular illnesses. A total of 79 GC patients were selected and split into two groups, namely nano carbon and control. Nano carbon suspension was employed to find and track LNs during surgery, and *ex vitro* anatomical LNs sorting was combined in the nano carbon group, whereas the control group used the traditional lymph node collecting approach.  Table 1 shows the general data of the two groups. This study was approved by the hospital ethics committee. All subjects gave informed consent and signed a complete informed consent form.

### 2.2. Application of Nano Carbon Tracer in Surgical LN Dissection

Usually, after the exploration, when the chief surgeon confirmed that the patients had no intra-abdominal and distant metastasis, the gastric tumor could be completely removed. Then, D2 radical operation was done in the control group to collect LNs. In the nano carbon group, nano carbon suspension (H20041829, Chongqing Laimei Pharmaceutical Co., Ltd., 1 mL: 50 mg) was adopted to locate the draining LNs around GC. After fully free exposure of gastric tumor, nano carbon suspension was injected at the edge of the lesion, and 4–6 points were selected for injection according to tumor's diameter. The injection volume of each point was 0.1–0.3 mL. After 1 mL tracer was injected within 3 minutes, the injection point was locally compressed with a gauze. To avoid injecting the tracer into the blood vessels, attention should be paid to reducing the inclination angle of syringe as much as possible. 10 minutes after tracer injection, the number and location of black LNs in the gastric cancer area were observed. Then, on the basis of D2 radical operation, the surgeon could carry out individualized dissection according to the black staining of LNs during operation.

### 2.3. *Ex Vitro* Anatomical LN Sorting

To further improve the detection rate of LNs in the samples, the lymph node sorting team was established to collect lymph nodes in the carbon nano group. The members were composed of 5 postgraduates in the department. Firstly, the team members need to be familiar with the anatomical knowledge of the stomach and then learn LNs location around the stomach and LN sorting method. Secondly, by observing the doctor's operation process, the team members observed the morphological characteristics of LNs *in vivo* and understood the corresponding tissues of LNs at each station in the separation process to combine the morphology of LNs *in vitro* and *in vivo*. Finally, improve the sorting members' ability to distinguish LNs (Figure 1). As LNs were often accompanied by vascular distribution, blood vessels in the specimen should first be identified in the sorting process, and then the adipose tissue along the blood vessels should be separated to better expose and obtain LNs. To avoid the missing of the smaller LNs, especially when the fat layer is thick, then it needs to be thinned layer-by-layer for separation. In terms of distinguishing LNs and fat particles, color and kneading with the index finger could be adopted. Generally, the fat particles are yellow. The color of LNs is relatively white, and the texture of LNs is relatively tough and not easy to crush. At each location, the collected specimens will be sorted into LNs and subsequently categorized for pathological analysis. LNs were sorted in the control group using traditional procedures. The two groups' LN metastasis was appraised and recorded following regular HE staining.

### 2.4. Indicators of Observations and Procedure for Evaluation

#### 2.4.1. Sorted LN's Number

In both groups, we have recorded both numbers, i.e., the total and micro, preferably in the sorted form, were noted. Additionally, the number of LNs, which are sorted at various infiltration stages along with different substations, were evaluated. These evaluations were performed to assess and ensure the total LN number (preferably in sorted form) in both groups.

#### 2.4.2. Total and Positive Number of LN's Correlation

The number of positive LNs in both groups was determined using HE staining data, and Pearson correlation exploration is utilized to determine the association of total and positive LN number, respectively.

#### 2.4.3. The Proportion of Black Stained LNs in LNs at Each Substation, Positive LNs, and Micro LNs

For the evaluation of the effect of nano carbon tracer in LN sorting, we compared the black staining in LN samples from different substations. Likewise, to examine the effects of the tracing of the nano carbon tracer in LN metastasis of GC, we have compared the black staining in positive LNs and micro-LNs.

#### 2.4.4. Clinical Treatment and Tumor Markers

In terms of intraoperative bleeding, the time of operation, postoperative exhaustion, postoperative feeding time, hospital stay, and postoperative complications, we compared the clinical management of the two groups. Furthermore, tumor markers can predict GC patients' prognosis and recurrence. CA199, CEA, and CA724 were chosen as GC's malignant biological signs in this investigation, and the levels of the above tumor markers were measured before and after surgery. EDTA was used to anticoagulate 5 mL venous blood samples. The supernatant was obtained after centrifugation at 1000 rpm and placed in the medical refrigerator at around 80°C for standby. ELISA was used to detect CA199, CEA, and CA724 levels. Abcam provided human CEA ELISA Kit (ab99992) and human CA199 ELISA Kit (ab108642), while Shanghai enzyme linked Biotechnology Co., Ltd provided human CA724 ELISA Kit (ml057569).

### 2.5. Follow-Up

We documented both the postoperative survival and recurrence rates of patients with various TNM stages to further investigate the influence of LN sorting on the prognosis of GC patients. WeChat, phone, and clinic were used to track down patients. The particular events of the disease progression, including as metastasis and recurrence, were the primary end point, whereas all-cause death was the secondary end objective. The term of follow-up concluded in January 2021.

## 3. Results and Discussion

### 3.1. Comparison of General Information of Both Groups of Patients

Both groups of patients had no remarkable differences in gender, age, BMI, etc., and they had comparability (Table 1).

### 3.2. More Total LN Number and Positive LN Number Were Sorted in Nano Carbon Group

By comparing the number of LNs sent for examination between both groups, the number in the nano carbon group was significantly more (Figure 2(a)), and so are the number of positive LNs (Figure 2(b)). Otherwise, more micro-LNs were detected in nano carbon group (Figure 2(c)). At the same time, we classified GC patients according to different invasion stages and different LN substations, and we found that the number of LNs sent for examination was more in the nano carbon group, and more positive LNs could be obtained (Figures 2(d)–2(f)). The above results suggested that obtaining more LN specimens was helpful to carry out more accurate clinical staging of GC to formulate a better follow-up treatment plan for patients.

### 3.3. Close Correlation Exists between Positive and Total LN Number

In the correlation analysis, we discovered a strong positive association between the total and positive LN numbers (Figure 3), signifying that for the detection of positive LNs, sort LNs are increased, which leads to an improved clinical staging accuracy.

### 3.4. Nano Carbon Suspension Is Helpful to Obtain LNs and Positive LNs

The lymphatic selectivity of nano carbon suspension helps to avoid its entry into the blood vessels to better show the drainage of regional LNs in GC. The obtained LNs were arranged according to the LN substation. The black-stained LNs obtained in N1 account for 62.02% of the total, and the black staining rates of LNs in N2 and N3 were 42.2% and 43.93%, respectively (Figure 4(a)). The above results suggested that nano carbon suspension could effectively label about 54% of the submitted LNs, which was helpful to improve the acquisition rate of LNs. Otherwise, nano carbon had a better black staining effect on LNs in the N1 station, which was conducive to the discovery of SLNs. While the black staining rate of LNs in N2 and N3 stations was similar, the black staining rate among micro-LNs was about 52.73% (Figure 4(b)), indicating that it was helpful to find and obtain more micro-LNs. In comparing the tracing effect of nano carbon suspension on positive LNs, it was found that 1326 black stained LNs were obtained in the nano carbon group, including 420 positive LNs, and 152 positive LNs were found in the nonblack stained group (figures 4(c) and 4(d)). The above results suggested that nano carbon suspension was helpful to obtain positive LNs.

### 3.5. The Clinical Treatment of Both Groups Was Similar, and Tumor Marker Level in the Nano Carbon Group Was Better Controlled

The clinical treatment of patients was evaluated from the aspects of the time of operation, time of postoperative exhaust, intraoperative bleeding, time of postoperative feeding, postoperative complications, and hospital stay (Table 2). The study showed that no obvious differences were found in the above indexes of both groups. Otherwise, the study found that the levels of CA199, CEA, and CA724 decreased more significantly in the nano carbon group (Figure 5), suggesting that the accurate clinical staging is helpful to formulate better follow-up treatment plans for patients to improve their prognosis.

### 3.6. Patients' Prognosis in the Nano Carbon Group Was Better

Patients were divided into I, II, and III stage groups according to the TNM stage, and their clinical prognosis was explored. In different clinical stages, the death risk and disease progression risk of patients in the nano carbon group were significantly reduced (Figure 6). The above results suggested that the increase of LN sorting number was helpful to the discovery of positive LNs to better evaluate patient's condition and take follow-up individualized treatment, thus reducing the risk of recurrence and death.

### 3.7. Discussion

During the GC therapy, an accurate clinical staging is the key point in the formulation of clinical plan and prognosis judgment [17]. Therefore, as an important part of GC clinical staging, improving the detection rate of positive LNs is the key problem to be solved in clinical treatment [18]. Previous guidelines have shown that the LN number detected during the operation should be greater than 16, which is a necessary condition for the accurate staging and prognosis evaluation, and the number of positive LNs detected is an independent risk factor for prognosis [19]. However, intraoperative LN collection will be restricted by many factors. In addition to the surgical resection method and the surgeon's clinical experience, obesity will greatly reduce the number of LN collection. Relevant studies have shown that the LN number harvested during an operation in GC patients with BMI greater than 27 is significantly lower than that in patients with BMI less than 25 [20]. Obesity will increase the difficulty of lymph node resection during operation and lymph node sorting after operation. In addition, the degree of tumor invasion is also an important factor affecting the collected LN number. With the increase of T stage, more lymph nodes can be collected in GC patients. In addition, micro-LNs are often missed in the process of surgery and sorting, however, about 40% of positive LNs belong to micro-LNs [14, 21]. Therefore, the missed detection of micro-LNs will bring adverse effects on the accuracy of TNM staging. To improve the detected LN number in GC patients, nano carbon suspension was used to label LNs, and LN sorting team was established to sort the isolated samples professionally.

Thanks to the unique lymphatic selectivity of nano carbon suspension, it can effectively display the LNs invaded by cancer cells around GC [22], which is important for the discovery of SLNs. Through the labeling effect of nano carbon suspension, it can guide doctors' operation methods and reduce surgical trauma. At the same time, it can also provide better reference for operators in LN dissection and improve the collection efficiency of LNs. Moreover, the professional sorting of isolated specimens after operation can effectively avoid the omission of LNs during operation, especially micro-LNs. Otherwise, by continuously summarizing the experience and optimizing the sorting process, sorting members can continuously improve the LN number. Therefore, the total number of LNs and micro-LNs obtained in the nano carbon group were significantly increased, and so has the total number of LNs obtained in different infiltration stages and lymph node substations. The number of positive LNs is important for appropriate staging since it is an independent risk factor for GC patients' prognosis. We discovered that the detection rate of positive LNs was higher in the nano carbon group and that the number of positive LNs was significantly correlated with the total amount of LNs detected, implying that if we increase the amount of sample collection of LNs, then it is highly likely that it can increase the rate of detection of positive LNs. Furthermore, in the carbon nano group, black-stained LNs account for 54.08 percent of total LNs and 52.73 percent of micro-LNs, with 31.67 percent of black-stained LNs being positive LNs, implying that the use of a nano carbon tracer can better assist doctors in collecting LNs and effectively improve the collection amount of positive LNs.

When the average number of LNs retrieved in GC patients is 25 or 40, Kim [23] discovered that the latter had a longer life time. Deng et al. [24] evaluated the clinical pathology data of 2455 GC patients and discovered that when the number of LNs increased, the TNM staging of the patients became more accurate, and their prognosis improved. The foregoing findings imply that in GC patients, there is a link between postoperative prognosis and harvested LN quantity. We discovered that in the nano carbon group, tumor indicators were better regulated, patients' conditions were more difficult to advance and relapse, and their mortality was lower. As a result, the increased number of sorting LNs will assist GC patients more.

## 4. Conclusion

In conclusion, nano carbon tracing combined with *ex vitro* anatomical sorting can effectively improve the detected LN number and the detection rate of positive LNs in GC patients. In particular, after the use of nano carbon tracer, black-stained LNs accounted for 54.08% of total LNs and 31.67% of positive LNs, respectively, which can assist doctors in better LN dissection and improve the collection of LNs. Otherwise, the number of positive LNs can improve the accuracy of clinical staging to optimize the further treatment plan after operation. Therefore, the level of tumor markers in the nano carbon group was better controlled and the prognosis of patients was better. However, some limitations exist in this study. The sample size of this study is small, retrospective analysis is easy to cause data bias, and there is no analysis and discussion on the relevant factors of LN detection, which needs to be improved in the follow-up study.

## Figures and Tables

**Figure 1:** Construction of *Ex Vitro* anatomical sorting system and LN sorting process.

**Figure 2:** Sorting of total LNs and positive LNs in both groups. (a) Comparison of total LNs. (b) Comparison of total positive LNs. (c) Comparison of micro-LNs. (d) Comparison of sorting LNs in different invasion stages. (e) Comparison of sorting positive LNs in different invasion stages. (f) Comparison of sorting LNs in different LN substations. ^*∗*^*P* < 0.05, ^*∗∗*^*P* < 0.01, and ^*∗∗∗*^*P* < 0.001.

**Figure 3:** Correlation analysis between the total LN number with positive LN number in nano carbon group (a) and control group (b).

**Figure 4:** Black staining of LNs in nano carbon group. (a) Number of black staining LNs in a different LN substation. (b) Number of black staining LNs among micro-LNs. (c) and (d) Comparison of positive LN number in black and nonblack staining LNs.

**Figure 5:** Tumor marker detection after surgery. (a) Serum CEA level detection. (b) Serum CA199 level detection. (c) Serum CA724 level detection. ^*∗*^*P* < 0.05, and ^*∗∗*^*P* < 0.01.

**Figure 6:** Analysis of the risk of death and disease progression. (a) and (b) Prognosis evaluation in GC patients with stage (I). (c) and (d) Prognosis evaluation in GC patients with stage II. (e) and (f) Prognosis evaluation in GC patients with stage III.

**Table 1:** General information table.

Factor	Nano carbon group (*n* = 40)	Control group (*n* = 39)	*F*	*P*
Gender			0.692	0.406
Male	31 (77.50)	27 (69.23)		
Female	9 (22.50)	12 (30.77)		
Age			2.062	0.151
≤50	14 (35.00)	8 (20.51)		
>50	26 (65.00)	31 (79.49)		
BMI (kg/m^2^)			0.485	0.486
≤23	28 (70.00)	30 (76.92)		
>23	12 (30.00)	9 (23.08)		
Tumor location			0.374	0.830
Upper 1/3 stomach	7 (17.50)	7 (17.95)		
Middle 1/3 stomach	11 (27.50)	13 (33.33)		
Lower 1/3 stomach	22 (55.00)	19 (48.72)		
Tumor diameter (cm)			1.360	0.243
≤5	26 (65.00)	30 (76.92)		
>5	14 (35.00)	9 (23.08)		
Radical gastrectomy			1.764	0.414
Proximal gastrectomy	2 (5.00)	4 (10.26)		
Distal gastrectomy	11 (27.50)	14 (35.90)		
Total gastrectomy	27 (67.50)	21 (53.84)		
Operation mode			2.318	0.128
Open surgery	19 (47.50)	12 (30.77)		
Laparoscope surgery	21 (52.50)	27 (69.23)		
Lauren typing			0.188	0.943
Intestinal type	13 (32.50)	14 (35.90)		
Diffuse type	19 (47.50)	18 (46.15)		
Mixed type	8 (20.00)	7 (17.95)		

**Table 2:** Recovery and clinical treatment.

Group	Cases	Operation time (min)	Intraoperative blood loss (mL)	Postoperative exhaust time (d)	Postoperative feeding time (d)	Length of stay (d)	Postoperative complications (%)
Nano carbon group	40	228.82 ± 30.24	44.34 ± 15.12	1.62 ± 0.73	4.76 ± 1.34	7.86 ± 3.78	3/40

Control group	39	238.38 ± 34.89	49.02 ± 13.43	1.89 ± 0.79	5.17 ± 1.43	8.42 ± 3.85	4/39
*t*/*χ*^2^		−1.302	−1.453	−1.578	−1.315	−0.652	0.186
*P*		0.197	0.150	0.119	0.192	0.516	0.666

## Data Availability

The dataset is available upon request.
